# Prevalence of gross lesions and handling practices in pigs and their association with pork quality, Kiambu, Kenya

**DOI:** 10.1371/journal.pone.0272951

**Published:** 2022-08-26

**Authors:** Derrick Noah Sentamu, Joshua Orungo Onono, Patrick Muinde, Nicholas Bor, Dorcas Chepyatich, Lian Francesca Thomas

**Affiliations:** 1 International Livestock Research Institute, Nairobi, Kenya; 2 University of Nairobi, Kangemi, Kenya; 3 World Animal Protection–Africa Office, Nairobi, Kenya; 4 University of Liverpool, Institute of Infection, Veterinary and Ecological Sciences, Liverpool, United Kingdom; Universidade do Porto Instituto de Biologia Molecular e Celular, PORTUGAL

## Abstract

Pre-slaughter handling of pigs has been documented to affect the quality of meat though no studies have investigated this relationship in the Kenyan context. This study aimed to determine the prevalence of gross lesions and practices related to sub-optimal welfare in pigs presented for slaughter while analyzing the relationship between occurrence of these lesions and meat quality. A cross-sectional study was conducted at a medium scale, non-integrated pig abattoir supplying to the Nairobi market, with a capacity to slaughter approximately 40 pigs a day. Data on welfare-associated lesions and handling practices were obtained from 529 pig carcasses and traders respectively. 387 pork samples were collected, and their quality evaluated by measuring their pH, meat color and drip loss. These three parameters were used to classify pork into four recognized categories namely: Red, Firm, Non-exudative (RFN), Pale Soft Exudative (PSE), Dark Firm Dry (DFD) and Red Soft Exudative (RSE). Almost all pigs were inefficiently stunned as evidenced by the presence of consciousness post-stunning. The majority of pigs (82.97%) having one or more welfare-associated gross lesions. Other animal welfare malpractices observed were high loading density and inadequate rest periods between transport and slaughter. A quarter of the pork samples were of sub-optimal quality including: RSE (11.36%), PSE (2.58%) and DFD (2.58%). Multinomial logistic regression revealed that pork originating from pigs transported at a high loading density had increased odds of being classified as DFD (OR 13.41, 95% CI 2.59–69.46). The findings indicate the need to educate stakeholders in the pork value chains on improved pig handling before and during slaughter to enhance pig welfare pre-slaughter and pork quality post-slaughter. Animal welfare legislation enforcement and implementation was observed to be insufficient. There is a need to educate key stakeholders on its importance of being put into practice both from economic and welfare perspectives.

## Introduction

Pork is a growing source of animal protein globally, the main producers being China and the European Union, with a steep upward trend in other regions of the world [1]. In Africa, pigs are increasingly contributing to improved nutrition and make a contribution towards household incomes, as they are relatively easy to rear and have a ready market [2,3]. The sub-Saharan African countries particularly Nigeria, Uganda, Malawi, Democratic Republic of Congo, Rwanda, Burundi, Ghana and Kenya have seen a rapid increase in the production and consumption of pork over the recent past [4]. The demand for pork in Kenya has been rising with the expanding and urbanizing human population with better incomes being a key driver. In 2012, approximately 129,450 tons of pork were produced in Kenya [5]. The demand for pork is predicted to increase by 268% between 2012 and 2050 [6]. The largest integrated pig slaughter facility in Kenya produces approximately 80% of the country’s processed pork products and exports approximately 2000 tonnes per year, while three less integrated and independent slaughter facilities located within Nairobi and multiple local slaughter slabs, all supply pork for the local markets [7]. The growth in the pig sector in the country is ongoing, yet with little attention paid to pig welfare [8].

Animal welfare refers to the physical and mental state of an animal in relation to the conditions in which it lives and dies. One construct of welfare considers the provision of five freedoms; the freedom from hunger and thirst, freedom from discomfort, freedom from pain, injury and disease, freedom to express normal behavior and the freedom from fear and distress [9,10]. On this basis, the Kenyan Prevention of Cruelty to Animals Act [11] clearly outlines the regulations to be followed in animal slaughter, and the penalties that have to be faced in contravention of this law. Efforts have further been made in enforcement of awareness on animal welfare in higher learning institutions like Universities and Technical schools offering animal sciences courses [12]. This step has provided a platform for non-governmental organizations (NGOs) and other bodies to join the welfare campaign.

Animal welfare also has economic implications on meat production. Inhumane treatment of animals during transportation and pre-handling before slaughter causes distress to animals [13]. Stress is defined as the physiological, behavioral and psychological state of the animal when confronted with, from the animal’s point of view, a potentially threatening situation [14]. This triggers the Sympathetic Nervous System and the Hypothalamic Pituitary Adrenal Axis to modify and release hormones that lead to physiological and metabolic responses [15]. These responses result in meat defects that include exudative pork: Pale Soft and Exudative (PSE) and Red, Soft and Exudative (RSE) pork; where glucagon hormone is released leading to a cascade of events. First it causes anaerobic breakdown of glucose, producing lactic acid that lowers muscle pH. This decreases the ability of muscles to hold water. Metabolic responses can also lead to Dark, Firm and Dry (DFD) pork where there is aerobic breakdown of glucose with no production of lactic acid, leading to high muscle pH and no breakdown of muscle fibers hence a lot of water is retained in the carcass postmortem [16]. The differing ultimate pH of pork from varying classes has been linked to increased microbial load within DFD and RSE meats, raising a potential food safety and food spoilage issue [17].

Several studies have reported associations between different pig management practices with welfare impact and pork quality categorization. For example prolonged fasting leads to PSE meat, unsuitable loading densities increases incidences of PSE and DFD pork, increased lairage time leads to DFD pork [17–20]. Therefore, “welfare practices” in this study also referred to the way pigs were handled by the different stakeholders.

There appears to be an increasing awareness by Kenyan consumers of animal welfare issues and a stated willingness to pay for improved welfare [12,21]. With an increasing middle-class with disposable income, demanding higher-quality animal source products, this indicates that pig welfare can no longer be ignored by the value chain stakeholders because consumers have been documented to be diverse and dynamic in their purchase behavior [22] and may boycott products which do not adhere to their demands.

Animal welfare is a relatively new field in Africa, with scarce data available on welfare issues across the continent [8,23,24]. To date, no studies on the influence of animal welfare practices on meat quality have been conducted in the Kenyan context. In Kenya there is a rise in intensive pig keeping with a market oriented approach and it is therefore important to understand how animal welfare is impacted in these value chains [2,5]. Kenya’s animal welfare and protection laws are also ranked as some of the best in Africa [25]. There is little data, however, on how these laws are enforced and baseline data such as that provided by this study identify areas where legislation and enforcement may require strengthening.

Science has an important role in underpinning societal decisions around animal welfare [26] and welfare assessments provide an evidence base as recommended by Blokhuis et al., [26], for enhancing compliance with and enforcement of animal welfare legislation. Observation of gross lesions and management-based practices are widely accepted approaches for assessment of animal welfare. Slaughterhouses are convergent points for animals and therefore important points for evaluation of animal welfare [12,27,28]. On this basis, this research aimed to determine the prevalence of gross lesions and handling practices related to sub-optimal welfare in pigs presented for slaughter and the relationship between the occurrence of these malpractices with technological meat quality. We hypothesized that a relationship between sub-optimal welfare and poor meat quality in this value chain may be present and that this data may be used to stimulate value chain actors to make animal welfare improvements in this value chain.

## Materials and methods

### Ethics statement

This study was approved by the International Livestock Research Institute, Institutional Animal Care and Use Committee (Ref no. 2019–36) and the Institutional Ethical Review Committee (ILRI-IREC2020-14), LFT holds a NACOSTI permit (NACOSTI/P/20/4847). Permission was also sought from both the National and Kiambu County Directorate of Veterinary Services and the slaughterhouse management. Informed consent to participate in the study was obtained from the person presenting each sampled pig for slaughter.

### Study site & sampling strategy

The target population for this cross-sectional study comprised of pigs raised for the urban terminus market, not including those pigs raised under contract for the one large fully integrated company present in the country. Between 5^th^ January and 5^th^ March 2021, we conducted this study at a medium scale, non-integrated pig abattoir located in Kiambu County, Kenya, with a capacity to slaughter approximately 40 pigs a day. The abattoir is open 6 days a week and therefore slaughters approximately 12400 pigs yearly. Kiambu County is located in the central region of Kenya and is the second most populous county (over 2.4 million people) according to 2019 Kenya National Bureau of Statistics Census report [29]. Kiambu County borders Nairobi and Kajiado Counties to the South, Machakos to the East, Murang‘a to the North and North East, Nyandarua to the North West, and Nakuru to the West. All these neighboring Counties combined have a population of over 10.7 million [29].

Kiambu County experiences bi-modal type of rainfall with long rains between Mid-March—May followed by a cold season usually characterized by drizzles and frost during June—August and the short rains between Mid-October to November. The average rainfall received by the county is 1,200 mm. The mean temperature in the county is 26°C with temperatures ranging from 7°C in the upper highland areas to 34°C in the lower midland zones. July and August are the months during which the lowest temperatures are experienced, whereas January—March are the hottest months. The County‘s average relative humidity ranges from 54 percent in the dry months and 300 percent in the wet months of March up to August [30].

All pigs presented for slaughter in the abattoir were eligible for sampling. An informed consent was obtained from the person presenting the pigs for slaughter. A minimum sample size of 384 pigs was calculated using a formula by Dohoo et al., [31] to detect a 50% expected prevalence of welfare associated gross lesions in pig, based on the lack of prior data on this prevalence, with a precision of 5% and confidence interval of 95%. Beginning with the first pig presented for slaughter after 6am on each sampling day, every 2^nd^ pig presented for slaughter was sampled. If the next pig to be selected according to the systemic random sampling originated from the same farm as a previously sampled pig, then this pig was ineligible for sampling and the next eligible pig was sampled and we returned to every 2^nd^ pig for the subsequent sampling. This sampling strategy ensured only one pig was sampled from pigs reported to originate from the same farm.

### Data collection

After obtaining informed consent from the person presenting the pig for slaughter, each recruited pig was weighed and data on its origin, date of purchase and method of transportation were entered into an Open Data Kit (ODK) (https://opendatakit.org/). As an abattoir procedure, each recruited pig was then directed into the stunning area by the abattoir workers. An ear tag was placed post exsanguination for ease of traceability. The loading space of the method of transportation and the number of pigs transported was used to calculate the loading density. Between the stunning area to the point of dispatch, data was collected and entered into an ODK form on handling practices and gross lesions which we believe *a priori* to be associated with sub-optimal animal welfare including;

- Observation of method of stunning & checking for presence of post-stunning consciousness signs immediately after stunning and prior to sticking, as described by Nielsen et al., [32] including; presence of tonic seizures, regular breathing, blinking and vocalizations.
- Observation for external and internal body lesions including; tether lesions which were scored as present or absent, tail bite lesions, loin bruising and hind limb bursitis as scored by Harley et al., [33]; skin lacerations and ear markings as scored by Bottacini et al., [34]; and pleuritis and pleuro-pneumonia as scored by Ceva & IZSLER, [35].

Pork samples were obtained from each carcass where the owner allowed us to sample and were collected according to the EZ-Drip Loss meat sampling procedure [36]. With the carcass hung on gambrels, immediately after splitting, a (9 x 7 x 2) cm^3^ meat sample was collected, always from the left-side silverside (*Biceps femoris*), after measuring horizontally from the highest point of the pubic bone, 13cm from the edge of the rind by the tail head. This was approximately 25 minutes after stunning in all cases, the meat samples were used to determine Drip Loss, pH and color. These samples were placed in a zip lock bag and kept in the cool—box for transportation to the laboratory at the department of public health pharmacology and toxicology, University of Nairobi for further analysis. Subsequent to the initial data collection period, the efficiency of stunning was followed up by measuring the amperage of the electrodes of the stunning device at the abattoir using 376 True-rms AC/DC Clamp Meter with iFlex™ [37].

### Laboratory analysis

In the laboratory, the lightness, pH and drip loss of the pork samples was evaluated. At an average room temperature of 18°C, the lightness (L*) of meat samples was obtained using a PCE–CSM 2 colorimeter (PCE Instruments UK Ltd, United Kingdom) with an aperture size of 8mm, a measuring angle of 45^0^ and a D_65_ illuminant. The device was calibrated daily before use as per the manufacturer’s instructions [38]. This involved placing a white calibration plate on the measuring aperture, followed by pressing the “Testing” button to start the calibration. A “Calibration Completed” confirmation display would appear on the screen after a few seconds. Pork samples were allowed to ‘bloom’ for one hour at room temperature as recommended by the American Meat Science Association (AMSA) [39] and Warriss [38]. Each sample was placed on a white background and the colorimeter measuring aperture placed on each to read in triplicates. The average L* value reading entered in an ODK form.

The ultimate pH (pH_24_) was obtained using a pH Meter FP20 (Mettler–Toledo, Switzerland) after storing the samples for 24 hours at 4°C. The device was calibrated daily before use. A two-point calibration was carried out where the electrode sensor was placed in calibration buffers of pH 4 and 7. De-ionized water was used to wash the electrode between measurements. The direct measurement of pH as described by Warriss [39] was used where the electrode sensor of the meter was inserted into the muscle tissue at different sites and the duplicate pH readings recorded in an ODK form. The average recording of the two readings was documented as the final pH of the meat.

The drip loss from the meat was obtained following the procedure outlined in the EZ-Drip Loss manual [36]. Within 6 hours of sample collection, two cylindrical portions (25ø × 25 mm) of each sample were obtained using the cylindrical knife provided in the kit. A drip loss container was weighed, and the weight recorded (W_C_). The bored cylindrical sample was then placed in the drip loss container, ensuring the meat did not contact the lid, and the combined weight of the meat and the container measured and recorded (W_T_). This was done in duplicate for all samples. The EZ-Drip Loss containers were then placed in the holder in the plastic box in the order they were sampled. The samples were kept upright in the container at 4°C for 24 hours. The meat sample was then removed from the drip loss container and the combined weight of the container, and the meat juice measured and recorded (W_1_). Drip loss was then calculated using the formula below.


EZ−Driploss=(W1−Wc)*100/(WT−WC)

Drip loss, pH and colour parameters were used to determine pork quality and their categories according to criteria by Warner et al., [40] as shown in Table 1.

**Table 1:** Classification of pork quality utilized in this study.

Quality Categories	pH24h	*Drip Loss %*	Color (L*)
PSE	< 6.0	> 5	>50
RSE	< 6.0	> 5	42–50
PFN & RFN	< 6.0	< 5	42–50
DFD	≥ 6.0	< 5	<42

#### Data management and statistical analysis

Data were collected using ODK and uploaded to the ILRI server every day after sampling and laboratory analysis. The datasets were later downloaded as.csv files, cleaned and merged for analysis in the R environment for statistical computing version 3.6.0 (2019-04-26) [41]. All lesions were collapsed into binary variables as present or absent. Descriptive statistics on prevalence of lesions and handling practices together with their 95% confidence intervals were calculated using the DescTools and gmodels package [42,43]. Loading density was calculated according to recommendations by Spoolder [44] based upon the weight of each pig. Both univariable and multivariable analyses were undertaken using the glmer function of the lme4 package [45].

Variables with p < 0.1 from univariable analysis were subjected to multinomial logistic regression using the multinom() function from {nnet} package and variables with a p-value less than 0.05 were considered significant (Assuming 5% significance level).

Acknowledging the potential confounding effect of transport type or loading density on both the presence of lesions and meat quality, it was determined that one or both of these variables would be retained in the final model. However, given that loading density is a derivative of method of transportation, and that only loading density had an association in univariate analysis, it was decided that between the two, loading density would be retained in the final model. Pigs from different farms being transported together (mixed batch) was also determined to be a potential confounder to the relationship between loading density and meat quality and was therefore retained in the final model.

The model was built backwards by gradually removing the less significant variables until a set of variables remained that produced the highest model accuracy, according to the lowest Akaike Information Criterion (AIC) value obtained. Possible model inaccuracy due to overfitting was addressed through cross validation where a train/test split was performed on the data.

## Results

Data was collected from five hundred and twenty-nine pigs (see Table 2) of which approximately half were female, and the mean live weight of the sampled pigs being 58.87 kg (range 13–230, SD 25.54) kg. The majority of pigs presented for slaughter at this abattoir originated from housed systems of Kiambu and Nairobi Counties. Others came from pig keeping counties in Central and Western Kenya (Homabay, Kajiado, Makueni, Murang’a and Nakuru Counties).

**Table 2:** Pig data as reported by those presenting pig to slaughter.

	Percentage count	Confidence Interval
**Sex**		
Male	46.2	41.89–50.57
Female	53.8	49.43–58.11
**Pig county of origin**		
Kiambu	79.58	75.79–82.91
Nairobi	12.72	10.04–15.96
Nakuru	3.08	1.83–5.07
Kajiado	2.7	1.54–4.60
Homabay	0.77	0.24–2.10
Makueni	0.77	0.24–2.10
Murang’a	0.39	0.07–1.54
**Husbandry system**		
Housed	97.8	95.87–98.74
Outdoor	2.32	12.62–41.34
**Pig presented by**		
Trader	86.32	82.99–89.10
Farmer	10.21	7.81–13.22
Middleperson	2.31	1.26–4.12
Butcher	1.16	0.47–2.62
**Transport means**		
Pick up	85.3	81.88–88.18
Motor bikes	7.16	5.15–9.82
Estate	2.9	1.69–4.85
Saloon	2.71	1.55–4.61
Tuk tuk	1.16	0.47–2.64
Bicycle	0.39	0.07–1.55
Walk	0.39	0.07–1.55

Pigs were transported to the slaughterhouse predominantly in pickups. Other means of transport were motor bikes (see Fig 1), bicycles, estate and sedan cars (see Fig 2), tuk tuks and walking. The mean loading density was 1.13 (95% C.I. 1.02–1.23, SD 1.06) m^2^/pig with nearly 1/3 of pigs transported at high loading densities as calculated according to methods by Spoolder [44]. Motor bikes had the highest mean loading density, 0.07 (95% C.I. 0.06–0.08, SD 0.03) m^2^/pig while “saloon” cars, which are sedans by design had the lowest mean loading density 2.11 (95% C.I. 1.58–1.05, SD 0.913) m^2^/pig (see Table 3).

**Fig 1:** An image showing a pig being transported using a motorbike.

**Fig 2:** An image showing a sedan vehicle for pig transportation.

**Table 3:** Summary on loading density by transport type.

Transport type	Mean m^2^/pig	Standard Deviation	Confidence Interval
Motor bikes	0.07	0.03	0.06–0.08
Bicycle	0.11	0	0.11–0.11
Tuk tuk	0.72	0.61	0.08–1.37
Pick ups	1.2	1.07	1.10–1.30
Probox	1.57	0.67	1.20–1.94
Saloon	1.58	0.91	1.05–1.58

The mean transport time for the sampled pigs was 1.23hrs (95% C.I. 1.15–1.31, SD 0.93) as estimated by those presenting the pigs for slaughter (range 0.5–10 hours). Approximately one fifth of the pigs were transported as a mixed batch with pigs from other holdings. Approximately half of all pigs were purchased, transported from the farm to the slaughterhouse, and slaughtered on the same day without any resting period.

A high proportion of pigs, 82.97% (95% C.I. 79.34–86.09%) had one or more gross lesions identified (see Table 4) with the most prevalent, being lacerations to the ears ‘ear marks’, utilized by traders to identify their pigs especially after scalding as the mark remains on the carcass (see Fig 3). Other gross lesions included: pleuropneumonia, tail bite lesions, tether lesions (mostly on the legs), loin bruising, lacerations, hind limb bursitis and liver milk spots. Head-only electrical stunning was utilized on all pigs, but a striking 99.61% (95% C.I. 98.43–99.93%) of pigs were inefficiently stunned as evidenced by post-stunning consciousness signs. An improvised handmade stunning device was used (see Fig 4) that was observed to be aged, corroded and dirty iron bars for electrodes (see Fig 5). This device was connected to direct current that fluctuated between 0.3–0.4 A and had a voltage of 245V. The stunning was done by different slaughterhouse operators who placed the tongs anywhere from the head to the base of the neck, for varying amounts of time which unfortunately we did not record. Subsequent to stunning, all pigs were bled using a heart stick, where long knives were deeply inserted on the ventral aspect of the base of the neck, just in front of the sternum.

**Fig 3:** An image showing an earmark on a pig, as made by slaughterhouse workers.

**Fig 4:** An image showing the improvised stunning device used in the study abattoir.

**Fig 5:** An image showing the dirty and corroded electrodes on the stunning device.

**Table 4:** Summary of gross lesions and practices observed.

Lesions and Practices	n/N*	Prevalence (%)	95% C.I.
Ear Marks**	373/484	77.07	73.00–80.69
Pleuro-pneumonia	94/344	27.33	22.75–32.42
Tail bite lesions	35/484	7.23	5.16–10.00
Liver Milk spots	22/459	4.79	3.10–7.28
Loin Bruising	20/484	4.13	2.61–6.42
Hind limb Bursitis	16/484	3.33	1.97–5.46
Tether Lesions	11/484	2.27	0.01–4.15
Lacerations	6/484	1.23	0.50–2.82
Electrical stunning	529/529	100.00	99.07–100.00
Incomplete stunning	510/512	99.61	98.43–99.93
Transported as mixed batch	103/511	20.16	16.82–23.95
Transported at high loading density	135/492	27.44	23.59–31.65
Purchase-slaughter interval > 24hrs	270/519	52.02	47.63–56.39

*due to the rapid nature of the slaughter process, we were not able to complete all observations for every pig hence N is variable for each observation

**Earmarks are lacerations made on the ears of pigs to enable identification by the traders. These marks are made with a sharp implement while the pig is still alive.

We were able to obtain 387 meat samples from pigs sampled in this study for analysis of technological qualities of meat. The collected meat samples were less than the number of pigs observed as not all individuals presenting pigs for slaughter were willing to sell a meat sample from their carcass, either due to their haste to leave the abattoir or desire to reap maximum revenue from the carcass despite consenting to providing a meat sample.

The majority of pork samples were classified as RFN, with 16.36% proportion classified as sub-optimal quality, being; RSE, DFD and PSE. The remaining samples could not be classified according to the quality criteria set for this study (see Table 5).

**Table 5:** Summary of technological meat quality attributes for all the categories of Pork.

		All samples	DFD	PSE	RSE	RFN
	No. Pigs (%)	387 (100)	10 (2.58)	10 (2.58)	44 (11.36)	184 (47.5)
pH_24_	Mean (SD)	5.61 (0.22)	6.27 (0.29)	5.48 (0.13)	5.52 (0.15)	5.57 (0.15)
	Range	5.17–6.92	6.00–6.92	5.37–5.76	5.27–5.94	5.17–6.00
Colour (L*)	Mean (SD)	44.28 (3.87)	39.44 (2.06)	53.17 (2.85)	45.58 (1.98)	45.29 (2.00)
	Range	35.23–59.48	35.23–41.48	50.05–59.48	42.04–49.36	42.05–49.75
Drip-loss (%)	Mean (SD)	3.10 (2.06)	1.45 (0.57)	6.79 (1.16)	6.86 (1.75)	2.55 (1.20)
	Range	2.89–3.30	0.61–2.30	5.49–8.70	5.02–11.98	0.00–4.97

SD–Standard Deviation

Univariate analysis between the classification of lesions and practices demonstrated some associations. These included: the time between purchase and slaughter, loading density and transporting pigs from different farms together as displayed in (Table 6). Transport type and loading density were associated (p < 2.2^−16^) and therefore transport type was excluded from further consideration in the model whilst loading density was retained.

**Table 6:** Variables demonstrating associations in univariate analysis.

	DFD 10	RFN 184	PSE 10	RSE 44	Total 248	p value
**Pigs transported** **with others from** **same farm only**						0.029*
• N-Miss	1	3	0	0	4	
• no	3 (33.3%)	33 (18.2%)	5 (50.0%)	14 (31.8%)	55 (22.5%)	
• yes	6 (66.7%)	148 (81.8%)	5 (50.0%)	30 (68.2%)	189 (77.5%)	
**Loading density**						0.002**
• N-Miss	1	8	0	1	10	
• Recommended	2 (22.2%)	133 (75.6%)	5 (50.0%)	31 (72.1%)	171 (71.8%)	
• High	7 (77.8%)	43 (24.4%)	5 (50.0%)	12 (27.9%)	67 (28.2%)	
**Purchase and** **Slaughter interval**						0.004**
• N-Miss	0	1	0	0	1	
• Slaughtered onpurchase day	6 (60.0%)	105 (57.4%)	6 (60.0%)	12 (27.3%)	129 (52.2%)	
• Slaughtered 24–48 hrs after purchase	4 (40.0%)	78 (42.6%)	4 (40.0%)	32 (72.7%)	118 (47.8%)	

* Represents significant variables. N-Miss means the number of missing observations.

Multinomial logistic regression demonstrated a negative association between purchase–slaughter interval and the meat quality classification in this study. Pigs slaughtered on the day of purchase had lower odds of producing RSE pork (OR 0.28, 95% CI 0.11–0.72). The study demonstrated a positive association between the loading density and the meat quality classification where transporting pigs at a high loading density was a risk factor for producing DFD pork (OR 13.41, 95% CI 2.59–69.46) (See Table 7).

**Table 7:** Variables included in the final multinomial logistic regression model with estimates of their coefficients, standard errors, odds ratios and confidence intervals of these odds ratios.

	Slaughter on day of purchase				High loading density				Pleuro-pneumonia				Transported as mixed batch			
	C	SE	OR	CI	C	SE	OR	CI	C	SE	OR	CI	C	SE	OR	CI
PSE	0.60	0.90	1.81	0.31–10.74	1.30	0.87	3.67	0.67–20.22	-14.87	953.00	3.50^−7^	7.4^−128^–3.17^+117^	- 0.70	0.93	0.50	0.08–3.09
DFD	0.49	0.77	1.63	0.36–7.44	2.60	0.83	13.41	2.59–69.46	-0.57	0.87	0.57	0.10–3.12	- 0.58	0.79	0.56	0.12–2.67
RSE	-1.26	0.48	0.28	0.11–0.72	0.60	0.50	1.81	0.68–4.84	-0.58	0.44	1.78	0.76–4.20	- 0.76	0.47	0.47	0.19–1.17
P-Value	0.02*				0.003**				0.06				0.39			

^**C**^ Coefficients, ^**SE**^ Standard errors, ^**OR**^ Odds ratios, ^**C.I**^ Odds Ratio Confidence Intervals Order followed for all variables.

*Represents significant variables.

## Discussion

This study reports the prevalence of welfare lesions and practices and their association with meat quality attributes in a porcine abattoir supplying pork to Nairobi city, one of the rapidly growing urban areas in Africa. We observed breaches in animal welfare during transport to the abattoir, in the identification of pigs (marking of ears with a sharp implement while alive) and stunning. Laboratory processing revealed that most of the meat were of sub optimal quality. A multivariate model demonstrated two associations between specific handling practices and sub-optimal meat quality.

Close to half of the pigs were reported to have been purchased directly from the farm, loaded and transported to the abattoir and slaughtered on the same day without being provided with resting time in the lairage to recover from the stressful processes of transport, loading and unloading. It is advisable to rest pigs for approximately 2–4 hours before slaughter in order to harvest good quality pork [46–48]. Resting also influences the pigs’ behavior and eases subsequent handling [49,50]. It should be noted that if pigs were transported or rested with pigs from different farms or rested in a lairage with these unfamiliar pigs resulted in fighting further stressing the pigs. Care should therefore be taken to address both the transport and lairage practices in this value chain simultaneously.

Transportation, by its nature, is an unfamiliar and threatening event in the life of an animal [51], and the over-crowding of animals further increases their stress levels. This study found that 27.44% of pigs were transported under conditions of high loading density violating the recommendations by Spoolder [44]. Such practice is commonly observed in the transportation of most animal species in Kenya [52]. This type of stress is known to cause elevated serum cortisol levels and can lead to hypoglycemia resulting in harvesting of DFD pork [53,54]. We found a positive association between high loading density and poor meat quality where an increase in loading density increased the likelihood of obtaining DFD pork. This type of pork has poor salability due to its dark-red appearance. DFD muscle fibers are depleted of stored glycogen, have high pH and tightly bind water. This enhances the muscles’ ability to absorb light as well as to avoid oxygen penetration, resulting into pork that appears dark red [54]. Our senses, for example sight, touch and smell are the first step in the process of assessing quality and freshness of meat before purchase [55] which is why this dark red appearance of DFD meat in a retail display has been reported as the leading cause of consumer rejection as they relate it to meat from old animals, spoilage, undesirable flavor, toughness, poor shelf life and staleness [56,57]. Additionally, insufficient acidification of DFD pork reduces its shelf life because high pH favors bacterial growth [16]. Besides being associated with harvesting sub optimal quality pork, high loading density can also lead to pig mortalities as observed by Ritter et al., [58].

Ideal transport conditions should allow pigs to stand or lie down [51] and the over-crowding of pigs during transport is against the Kenyan Prevention of Cruelty to Animals (Transport of Animals) Regulations [59] Regulation 8 which states that “*The transporter or other person in charge of animals transported in vessel*, *aircraft or vehicle*, *or any pen therein*, *shall ensure that the animals are not overcrowded and are so accommodated as to avoid any risk of injury or unnecessary suffering*. *A person who fails to comply with this Regulation shall be guilty of an offence*.” These inhumane methods could be as a result of lack of awareness that pigs are sentient beings, lack of knowledge on recommended loading densities and generally about animal welfare as deduced by Descovich et al., [60] in China. This challenge was also reported by welfare advocacy organizations in Africa in a study by Tan [24], where they described that such challenges are maintained because animals are commonly regarded as food, tools and commodities unable to process positive or negative experiences and not worthy of moral consideration if they will be slaughtered anyway. The trend of livestock intensification in Africa is also a possible cause as it comes with commercial pressures that lead to tradeoffs in animal welfare for profit maximization [61].

We observed transportation of pigs to the abattoir using inappropriate means such as packing them into sacks and loaded onto motor bikes and bicycles, although at a lower level than reported in rural western Kenya (88%) where this method of transportation is the norm [62]. Dependency on motorbikes for pig transportation to this abattoir has previously been reported as a challenge by pig traders [7], who further explained that motor bikes are a solution to the high cost of transportation. Masiga and Munyua [52] also explained that motor bikes are used due to lack of specialized vehicles for animal transport. Wambui et al., [63] came to a similar conclusion, that there were no vehicles dedicated for transportation of livestock in Kenya. As much as use of non-specialized transport may be convenient and cheap, it undermines the welfare of pigs by exposing them to the potential for fractures and other injuries and even mortalities and contravenes the Prevention of Cruelty to Animals (Transport of Animals) Regulations [59] Regulation 8. Kenyan law states that vehicles transporting pigs ought to have good ventilation systems to avoid heat stress to the pigs, good suspension to avoid excessive vibrations that can cause muscle fatigue, non-slippery floors to avoid falls and the structure of the sides ought to be smooth without protrusions and sharps to avoid injuries. Detailed recommendations on vehicle designs suitable for transportation of pigs are given by Spoolder, [44] and FAO, [64].

Our study found that 77.07% of the pigs were marked on the ears with knives by slaughterhouse workers, where initials of the names of the owners were inscribed deep into the ears for identification and follow-up in the slaughter line. Ear marking causes injury to the animal and according to the description of Sanni [65] this could be abuse of animals due to ignorance. Similar practices, based on the same rationale, have been reported in Italy and Uganda [34,66]. Such an identification method is probably used because of the dearth of well-established identification systems in the nation, with less technical solutions being more feasible [8]. This practice violates OIE, [10] recommendations that animals must be free from injury and pain. With humane restraint, other possible affordable and less invasive alternatives to this practice include: scrapping off bristles of pigs still with sharp blades to form signs unique to each owner as practiced in Nigeria [67] and use of slap marks as practiced in the United Kingdom [68].

Almost all animals in our study (99.61%) showed signs of consciousness after stunning, presence of which indicates that the stunning was ineffective [32]. Several factors exist which may have contributed to this observation, these include: Head only electrical stunning on unrestrained animals, poorly made electrode set and fluctuating electrical current and improper placement of electrodes. Such practices also elicit pain and fear and compromise welfare [69]. Ideally, stunning should render the pig instantaneously unconscious, long enough until bleeding results in enough loss of blood to cause death from lack of oxygen to the brain [70,71], in the absence of this there will be persistence of consciousness in the subsequent steps of the slaughter process [32]. The stunning was executed using a V–shaped handheld device with electrodes on each side, similar to that described by Spencer & Veary, [72] in South Africa. These electrodes, however, were tied together on either side of a piece of wood that served as a handle and was connected to direct current. This means current flowed through the electrodes continually during the stunning process and this is a potential hazard to the abattoir workers. Contrary to recommendations on tong maintenance by FAO [64], the electrodes were old, corroded and appeared un-cleaned and poorly maintained which is a potential cause for ineffective stunning through electrical impedance [73]. There was no fixed position of the tongs on the animal while stunning and these were placed anywhere from the head to the base of the neck, (see Fig 6), a similar finding to [74], contrary to the ideal placement of electrodes recommended by Anil & McKinstry [69] under field conditions. For current to reliably pass through the brain while using head only electrical stunning, the electrodes should be placed against the base of the ears.

**Fig 6:** An image showing how the stunning device was placed while stunning.

Wrong placement of electrodes was further aggravated by a low amperage system that delivered an electric current that fluctuated between 0.3–0.4 A. The voltage to the device was 245 – 248V but due to a high electrical resistance, probably as a consequence of the improvised design and poorly maintained state of the device, the ultimate current dispensed to stun the pigs was very low, way lower than the recommended 1.3A, the least current required to induce a grand mal epileptic seizure, during head only electrical stunning for pigs [32,47]. Using such low electric current risks the pigs experiencing a painful electric shock before onset of unconsciousness [73]. Other possible reasons for ineffective stunning could be lack of knowledge of slaughterhouse workers on the purpose of stunning with regards to animal welfare and lack of training on proper execution of the practice. Ineffective stunning could also have been due to the unsuitable design of the stunning area. It had limited space shared between one stunning personnel, several pigs and other slaughterhouse activities, contrary to guidelines for head only electrical stunning for pigs without restraint, which recommend at least 2 operators and 1.2m^2^/pig space allowance in the stun pen [47]. All these contravenes Section 8 of the Kenyan Prevention of Cruelty Act [11] that states *“Any person who*, *whether in any slaughterhouse or abattoir or in any place than a slaughterhouse or abattoir*, *and whether for human consumption or not*, *slaughters an animal—(a) in such a manner as to cause it more suffering than is necessary; or (b) in the sight of any another animal awaiting slaughter*, *shall be guilty of an offence and liable to a fine not exceeding two thousand shillings or to a term of imprisonment not exceeding three months or to both*.*”*

In the event that the V–shaped stunning device has a proper design, well maintained electrodes and therefore a sufficient amperage, head/heart electrical pig stunning method as recommended by Vogel et al., [75] could be a proper working alternative to head only electrical stunning. This is a 2-stage stunning method where head-only stunning for 3s is immediately followed by application of the same stunning device to the cardiac region for 3s, while the animal is lateraly recumbent. Head/heart electrical stunning renders the pig unconscious for a longer period compared to head only electrical stunning. This longer interval creates sufficient time to carry out bleeding while the animal is completely unconscious, allowing for compliance with humane slaughter regulations. It is also important to note that because of pigs maintaining consciousness even after stunning, inhalation of blood into the lungs at exsanguination was observed (see Fig 7). Such lungs could present quality challenges for small businesses that sell them as food and for entrepreneurs that further process them into other products.

**Fig 7:** An image showing a congested lung.

A key finding of this study of relevance to the sustainability and profitability of this value chain was that 16.6% of pork samples tested in this study were found to be of sub-optimal quality with 13.94% (95% C.I. 10.74–17.90%) being of an exudative type (RSE & PSE). Excessive exudates from meat have been associated with microbial spoilage [76]. Drip loss can also be a major source of food wastage and financial losses [77]. According to our study, the mean drip loss for the exudative categories of pork were 6.79% and 6.86% for PSE and RSE respectively in comparison to the 2.54% for optimal quality meat. This indicates that for every kg of pork, RSE pork loses an additional 43.2g compared to optimal (RFN) pork, in 24hrs. At the current market price of 320 Kenyan Shillings per kg, this amounts to a potentially additional daily loss of Kshs 13.82 (0.13 USD) per kg, compared to optimal quality meat. With the multiplier effect, (across multiple carcasses) these are substantial losses to stakeholders in this pork value chain. This is in agreement with a study by Juliet et al. [77] in Uganda where drip loss was found to be the second major cause of beef losses, together with meat wastage (drops of meat and bones that fall off during cutting of beef for sale) where the two factors led to losses of up to 787.50 USD daily per district of study.

Besides potential loss of income due to exudative meat, other losses result from decreased willingness to pay by the consumers for poor looking meat. Otieno & Ogutu [22] carried out a study on consumer willingness to pay for chicken welfare attributes in Kenya and found that chicken consumers in Nairobi had a positive and significant preference for use of certified transportation means, humane slaughter of chicken and animal welfare labeling of chicken. AU-IBAR [12] reported that Kenyan pork consumers have made inquiries to pig slaughter–houses on good animal welfare products. Consumers have also increasingly expressed a lack of faith in food quality and control systems, yet it’s an important factor in their purchase decision [57].

Therefore, this is not only indicative of increased awareness and concern towards animal welfare and sentience by the Kenyan meat consumer, but also of the unexplored financial benefits that may come with improvement of the same. Fernandes et al. [78] stresses that improvement of perceived product quality is a benefit to businesses, therefore addressing the welfare aspects highlighted by this study has the potential to yield more income. Asmare [79] also notes that there is a steadily emerging global trend of consumer requirements dictating product qualities and specifications, this further stresses the need to improve pig welfare given the growing concern of Kenyan consumers regarding animal welfare.

Kenya has dedicated animal welfare legislation, the Prevention of Cruelty to Animals Act (1983) [11] which is one of the most comprehensive and inclusive pieces of legislation on animal welfare issues in Eastern Africa and defines what constitutes an animal cruelty offence and the subsequent penalties [52]. Kenya is also in a unique position with the currently tabled Animal Welfare and Protection Bill [80] that has detail on observation of animal welfare in the nation and the Draft National Livestock Policy [81] that acknowledges animal welfare as an important concept. However, with this legal arsenal in place, it leaves a lingering question on why there is inadequate enforcement and implementation, a challenge/weakness also acknowledged by AU-IBAR [12] in their assessment of animal welfare in the East African nation. This challenge highlights the need for political will in the advocacy of animal welfare, which has been shown to be successful in other countries including Ecuador and Chile [82]. Political will is the commitment of political leaders and bureaucrats to undertake actions to achieve a set of objectives and to sustain the costs of those actions over time, resulting in sufficient allocation of human and financial resource to effectively enforce the laws that they make [83].

Insufficient legislative enforcement of animal welfare issues undermines efforts to improve animal welfare. It is therefore important to develop creative solutions to address this challenge. For example, animal welfare advocacy organizations could capitalize on political engagement concerning legislative enforcement [52]. Ngwili et al. [84] emphasizes that effective solutions and future interventions to society challenges, in this case poor animal welfare, should be underpinned by baseline studies to understand their contextual factors and enabling environments. These may be socio-economical, anthropological, environmental, cultural, geographical or even political factors. Understanding context in which sub-optimal animal welfare thrives, will help design interventions to improve practices and to educate the public about the importance of good animal welfare [85].

This study had a few limitations. Due to the rapid nature of the slaughter process, we were not able to complete all observations for every pig and some of the traders who had consented for their pigs to be included in the study later were unwilling to sell a meat sample to us. For that reason, observational data from 142 pigs did not have corresponding meat samples. Whilst we do not believe there was any systematic bias in this refusal to sell a meat sample and that it likely stemmed from the rapid nature of the process and a desire in the trader to quickly process the carcass to sell, it could be hypothesised that traders who believed there to be a problem with their meat to be more likely to refuse to allow the sample to be taken.

The study also echoes the need for more animal welfare related studies for example, consumer preference and willingness to pay as influenced by technological quality attributes of harvested meat, knowledge, attitude and practices concerning animal welfare legislation, stunning and transportation practices.

## Conclusion

This study was one of the first studies on meat quality and animal welfare for pigs in Kenya, documenting practices that breach animal welfare, including: poor means of transportation, mixing pigs of different farms during transportation, transporting animals at high loading densities and immediate slaughter of animals without adequate rest. The study also observed a high prevalence of welfare associated gross lesions with labels made on ears using sharp objects being the most prevalent. We observed that nearly all the pigs were poorly stunned as indicated by the presence of consciousness signs post stunning. A high prevalence of poor-quality pork especially the exudative type was also observed. These findings are indicative that pre–slaughter handling of pigs is capable of affecting the quality of harvested pork and that this plays into the intricacies of consumer preferences and ultimately the salability of the final product. We have seen that animal welfare legislature is present in the country but there is inadequate enforcement and adherence to it, highlighting that law enforcement authorities and other legal entities tasked with safeguarding animal welfare need to improve their practices. We highly recommend slaughterhouse personnel are provided with basic animal welfare training, including; appropriate handling of live animals, humane identification techniques and on efficient head-only electrical stunning to urgently improve the animal welfare situation in the country and to improve the economic efficiency of the industry.
